# TSTELM: Two-Stage Transfer Extreme Learning Machine for Unsupervised Domain Adaptation

**DOI:** 10.1155/2022/1582624

**Published:** 2022-07-18

**Authors:** Shaofei Zang, Xinghai Li, Jianwei Ma, Yongyi Yan, Jiwei Gao, Yuan Wei

**Affiliations:** ^1^College of Information Engineering, Henan University of Science and Technology, Luoyang 471000, China; ^2^College of Vehicle and Traffic Engineering, Henan University of Science and Technology, Luoyang 471000, China

## Abstract

As a single-layer feedforward network (SLFN), extreme learning machine (ELM) has been successfully applied for classification and regression in machine learning due to its faster training speed and better generalization. However, it will perform poorly for domain adaptation in which the distributions between training data and testing data are inconsistent. In this article, we propose a novel ELM called two-stage transfer extreme learning machine (TSTELM) to solve this problem. At the statistical matching stage, we adopt maximum mean discrepancy (MMD) to narrow the distribution difference of the output layer between domains. In addition, at the subspace alignment stage, we align the source and target model parameters, design target cross-domain mean approximation, and add the output weight approximation to further promote the knowledge transferring across domains. Moreover, the prediction of test sample is jointly determined by the ELM parameters generated at the two stages. Finally, we investigate the proposed approach in classification task and conduct experiments on four public domain adaptation datasets. The result indicates that TSTELM could effectively enhance the knowledge transfer ability of ELM with higher accuracy than other existing transfer and non-transfer classifiers.

## 1. Introduction

In the current era of big data, the classification model constructed by machine learning can help human quickly identify and annotate a large number of images, texts, audios, and signal data rapidly generated by the Internet, sensors, and computers. Mining information from these data helps understand the relationship between things. Support vector machine (SVM) [1], k-nearest neighbor (kNN) [2], naive Bayes [3, 4], decision tree [5], logistic regression [6], and many other classifiers with high accuracy appear and have attracted much attention. Huang et al. [7] proposed extreme learning machine (ELM) which is a better classifier with powerful nonlinear fitting and approximation capabilities [8, 9] and has been widely studied and applied in brain-computer interfaces [10, 11], medical diagnosis [12, 13], fault diagnosis [14], hyperspectral [15], and other fields.

ELM initializes randomly the input weight and bias and obtains optimal output weight by solving a least-squares problem [7–9, 16], which has the advantages of faster learning speed and better generalization, therefore becomes a hot research topic. There are many variants of ELM put forward both in theories and applications to enhance its performance for handling problems in different situations. In order to solve the problem that ELM is sensitive to the input weights and biases, Li et al. [17] proposed a WOA-ELM algorithm which applied the whale optimization algorithm (WOA) to optimize the input weights and biases of ELM for its performance improvement. In response to the class imbalance problem, weighted extreme learning machine (WELM) [18–20] was proposed, in which different weights are assigned for each training sample based on two different strategies. SMOTE based on class-specific extreme learning machine (SMOTE-CSELM) [21] was also presented by exploiting the benefit of both the minority oversampling and the class-specific regularization. To improve the generalization power and prevent the overtraining of ELM, some methods combined ensemble learning with it to improve its robustness, including voting-based extreme learning machine (V-ELM) [22, 23], AdaBoost extreme learning machine [24–26], and extreme ensemble of ELMs (EEoELMs) [27]. Moreover, affected by deep learning, ELMs with deep structure occur for high accuracy. ML-ELM [28, 29] was presented to resolve the time-consuming issue of deep learning and achieved faster speed and higher generalization than stacked autoencoders, deep belief network, and deep Boltzmann machine. Hierarchical ELM (H-ELM) [30, 31] was proposed to enhance the universal approximation capability of ELM. The kernel-based multilayer ELM (ML-KELM) [32] integrated the kernel learning technique into the ML-ELM and achieved a faster learning speed and a better recognition performance. Although the above ELM models have achieved great success in classification and regression tasks, they will degrade when training samples and test samples are taken from different domains with different distributions (i.e., cross-domain tasks).

To handle this problem, domain adaptation (DA) [33–35], as an important branch of transfer learning, has attracted wide attention, in which efficient classifier is obtained with the help of the knowledge from source domain, which is different but related to target domain. L. Zhang and D. Zhang [36] put forward the domain adaptation extreme learning machine (DAELM) framework by extending ELM to handle domain adaptation problems for gas identification and drift compensation of E-nose system. Adaptive ELM (AELM) [37] was proposed by introducing the manifold regularization term into ELM for image classification. Zang et al. [38] proposed a supervised extreme learning machine called transfer extreme learning machine with output weight alignment (TELM-OWA), which aligned the output weight matrix of the ELM between domains and added the approximation between the inter-domain ELM parameters for knowledge transferring. However, these approaches are developed to solve semi-supervised domain adaptation problems because they require few labeled samples from the target domains. Due to its high cost in collecting labels and labeling samples, cross-domain ELM (CDELM) [39], domain space transfer ELM (DST-ELM) [40], cross-domain extreme learning machine (CdELM) [41], and extreme learning machine based on maximum weighted mean discrepancy (ELM-MWMD) [42] are proposed respectively for unsupervised domains by minimizing the classification loss and applying the maximum mean discrepancy (MMD) strategy on the prediction results. In the above methods, the supervised ELM model usually outperforms the unsupervised ones with the help of a few labeled samples from the target domain.

In this article, inspired by pioneering works [38, 42], we propose a novel method denoted as two-stage transfer extreme learning machine (TSTELM), in which there are two stages of domain adaptation: statistical matching and subspace alignment. At the statistical matching stage, we first learn a domain adaptation ELM classifier via utilizing the MMD to simultaneously minimize the marginal and conditional distribution between domains. In addition, at the subspace alignment stage, we use a transformation matrix to align the output weights of inter-domain ELM models, simultaneously put forward target cross-domain mean approximation, and add an output weight approximation term into the objective function. Then we can obtain the other domain adaptation ELM. Finally, we fuse the DAELM parameters from two stages to realize the label prediction of test samples. TSTELM is illustrated in Figure 1. Extensive experiments have been conducted on real-world image and text datasets, and the results verify that our approach outperforms several existing domain adaptation and non-domain adaptation methods.

In this article, TSTELM realizes knowledge transferring at two stages, and its contributions are summarized as follows:

1. Similar to [39], our method is to use MMD proved as a general statistical distribution discrepancy measure, to minimize the marginal and conditional distribution discrepancy of the outputs of hidden lays of ELMs from two domains, which effectively extends ELM for unsupervised domain adaptation. Therefore, we can obtain one DAELM.
2. Based on the first DAELM and inspired by [42], we introduce the output weight alignment, design target cross-domain mean approximation, and add the output weight approximation constraint into traditional ELM for enhancing knowledge transfer across domains. Hence, we can learn the other DAELM. It is worth emphasizing that we present target cross-domain mean approximation referred to [35] to adapt the distribution of the target domain for consistency with the source domains.
3. At prediction stage, the above two DAELMs jointly determined the category of test samples. Our proposed method performs image classification experiments on object recognition and text datasets. The results verify its effectiveness and advantages.
4. Compared with other the state-of-the-art DAELMs, our research has some distinct properties: (1) Many technologies including MMD, output weight alignment, output weight approximation, and target cross-domain mean approximation are utilized to jointly realize the efficient knowledge transfer across domains at two stages. (2) Output weight alignment organically bridges the DAELMs from the statistical matching stage and subspace alignment stage. (3) Joint decision from two DAELMs facilitates our approach to obtain robustness and high accuracy.

The rest of this article is organized as follows: In Section 2, we briefly review domain adaptation and ELM. We then present the proposed TSTELM in Section 3. In Section 4, the experiment and analysis are presented. Finally, Section 5 is the conclusion of this article.

## 2. A Brief Review of the Domain Adaptation and Extreme Learning Machine

### 2.1. Domain Adaptation

When the training and testing data are drawn from different distributions, a classifier directly learned on training data would have a poor performance for testing data. Domain adaptation is developed to deal with this scenario, in which an excellent classifier could be obtained from the source domain with rich labeled samples and perform well in the target domain task. The source domain and the target domain have different distributions but some correlations.

In the past decades, many researches have conducted to address domain adaptation problems in classification task, which are mainly divided into three parts [35, 43]: (1) Sample-based adaptation. It directly assigns weights to each sample of two domains, which could adapt and minimize the distribution gap between domains. Many such approaches appeared such as domain adaptation (PRDA) [44], TrAdaBoost [45], and Kernel Mean Match (KMM) [46]. (2) Feature-based adaption. It seeks the shared subspace between domains, in which distribution discrepancy is alleviated and knowledge is easily transferred across domains. Transfer component analysis (TCA) [47] and joint distribution adaptation (JDA) [48] take MMD metric as an objective function to find an optimal projected matrix for shared low-dimensional subspace. Liang et al. [49] designed a relaxed domain-irrelevant class clustering (DICE) term and then combined it with MMD to obtain a domain-irrelevant projection for reducing distribution discrepancy between domains. Moreover, DICE was extended to ensemble learning with multiple projection obtained from sampling subsets of source and target domains, which help it achieve better performance. Progressive learning with Confidence-wEighted Targets (PACET) [50] improved DICE by adding a confidence-weight strategy with the posterior probability of target instance. (3) Classifier (or parameter-based) adaptation. Its purpose is to find optimal classifier or its parameter with a well-generalized ability between the source and target domains. Yang et al. [51] presented adaptive support vector machine (Adapt-SVM). It designed a regularizer to minimize the discrepancy between parameters of two classifiers trained on source and target labeled samples and then added into SVM's objective function. Multi-model knowledge transfer (Multi-KT) [52], following the idea of Adapt-SVM, constructs a regularizer to force the parameter of target SVM close to multiple weighted source SVMs. In multiple kernel learning, Wang et al. [53] introduced multiple kernel MMD into the objective function to adapt distribution discrepancy between training samples and test samples, which prevents performance degradation because of inconsistent distribution of datasets and simultaneously obtain a multiple kernel classifier with strong generalization ability. Recently, deep network adaptation and adversarial learning adaptation have become successful in computer version and machine learning. Based on the assumption that samples with the same category are close each to other and the local geometry property of the data can be maintained in neural embedding subspace, Wang et al. [54] proposed the neural embedding match (NEM), which reduces cross-domain distribution divergence by projecting the source and target domains into a common subspace using deep neural network embedding model. In [55], a deep neural network with weighted MMD and the manifold embedding was proposed to handle domain adaptation for hyperspectral image classification. To address the problem in unsupervised partial domain adaptation (PDA), Liang et al. [56] put forward a domain adversarial neural networks called BA^3^US. It presented balanced adversarial alignment (BAA) and adaptive uncertainty suppression (AUS) to overcome negative transfer and propagation of uncertainty which usually appear in PDA.

In the abovementioned approaches, sample-based adaptation methods are the most efficient ones for knowledge transfer because of direct utilization of source sample, while feature-based adaptation methods are widely applied. Classifier (or parameter)-based adaptation is the most potential one due to past related domain knowledge or experience is integrated into shared parameters of classifier. Deep network adaptation and adversarial learning adaptation strictly belong to feature-based adaptation method but they can extract (deep) domain-invariant feature with strong discrimination. However, these methods also have their own shortcomings. In sample-based adaptation methods, the effective evaluation mechanism about sample importance is a challenge. Generic shared features obtained from different domains is also a difficult task in feature-based adaptation methods. Since the useful information and knowledge from the auxiliary domain to the target domain is not directly applied, classifier (or parameter-based) adaptation is not efficient compared with two formers. Deep network adaptation usually needs massive labeled samples and sufficient computing resources for training deep model, which could hinder its application. Class misalignment and the simultaneous efficiency of feature extractor and discriminator are a challenge for adversarial learning adaptation. In this article, our approach belongs to classifier (or parameter)-based adaptation; it attempts to seek two output weights of shared ELM models across domains for knowledge transferring.

In this article, we propose TSTELM to address problems in the unsupervised domain adaptation, in which the training data come from the source domain with labeled samples and the test data come from the target domain with unlabeled samples. Suppose the source domain dataset is denoted as {(**x**_*Si*_, **y**_*i*_)}_*i*=1_^*n*_*S*_^ ∈ **D**_*S*_ and the target domain dataset is denoted as {(**x**_*Tj*_)}_*j*=1_^*n*_*T*_^ ∈ **D**_*T*_, where *n*_*S*_ and *n*_*T*_ represent the number of source and target samples, respectively. The source data and the target data belong to the same feature space *𝒳*_*S*_=*𝒳*_*T*_ and label space *𝒴*_*S*_=*𝒴*_*T*_. The data distributions of the source and the target domains should be different but similar, that is the marginal distribution *P*(**X**_*S*_) ≈ *P*(**X**_*T*_) and conditional distribution *P*(**Y**_*S*_*| ***X**_*S*_) ≈ *P*(**Y**_*T*_*| ***X**_*T*_). In TSTELM, we hope to construct an ELM model using {(**x**_*s*(*i*)_, **y**_*s*(*i*)_)}_*i*=1_^*n*_*S*_^ to obtain high accuracy on {**x**_*Te*(*k*)_}_*k*=1_^*n*_*Te*_^. Table 1 summarizes other related notations in domain adaptation problems.

### 2.2. Extreme Learning Machine

Unlike the conventional feedforward neural networks, ELM is an approach in which two characteristics are contained: (1) Hidden layer parameters (i.e., input weights and the biases) can be randomly initialized. (2) The output layer weight can be solved as the least-squares problem. As a result, it yields faster learning speed and better generalization performance compared with other classifiers.

Given a training set {(**x**_*i*_, **y**_*i*_)}_*i*=1_^*N*^ with *N* samples, where **y**_*i*_ is the label corresponding to **x**_*i*_, and **C** is the number of categories. The structure of the ELM with *L* hidden nodes and activation function *h*(*x*) is shown in Figure 2:

In Figure 2, *x*_*i*_ is the input sample, **w** is the input layer weight, **b** is the hidden layer bias, and the hidden layer output *h*(*x*) is calculated as: *h*(*x*_*i*_)=*g*(**w***x*_*i*_+**b**). Here, *g*(*x*) is the nonlinear activation function, *L* is the number of nodes in the hidden layer, and *β*_*i*_ is the hidden layer output weight. The outputs of the network are given by:

(1) $$\begin{array}{c} y_{j}=\sum_{i=1}^{L}\beta_{i}h\left(w_{i}\cdot x_{j}+b_{i}\right),j=1,2,\ldots ,N. \end{array}$$

The above formula can be written in matrix form:

(2) $$\begin{array}{c} Y=\mathrm{H\beta}, \end{array}$$

where $H={\left[\begin{array}{ccc} h\left(w_{1}\cdot x_{1}+b_{1}\right) & \cdots & h\left(w_{L}\cdot x_{1}+b_{L}\right)\\ \vdots & \ddots & \vdots \\ h\left(w_{1}\cdot x_{N}+b_{1}\right) & \cdots & h\left(w_{L}\cdot x_{N}+b_{L}\right) \end{array}\right]}_{N\times L},\beta =\left[\begin{array}{c} \beta_{1}\\ \vdots \\ \beta_{L} \end{array}\right],\text{ and }Y=\left[\begin{array}{c} y_{1}\\ \vdots \\ y_{N} \end{array}\right]$_._

By adopting parameter regularization, the ELM can avoid the overfitting problem. Its corresponding objective function can be formulated as

(3) $$\begin{array}{c} \underset{\beta }{\min}L_{\text{ELM}}=\frac{1}{2}{\left\|\beta \right\|}^{2}+\frac{\theta }{2}{\left\|Y-\mathrm{H\beta}\right\|}^{2}, \end{array}$$

where *θ* is a penalty constant on the training errors, and ‖•‖^2^ denotes the L2-norm of a matrix or a vector.

The minimization of equation (3) is a regularized least-squares problem. By setting the gradient of equation (3) with respect to *β* as zero, we have

(4) $$\begin{array}{c} \nabla L_{\text{ELM}}=\beta +\theta H^{T}\left(Y-\mathrm{H\beta}\right)=0. \end{array}$$

The output weight vector *β* is obtained according to the Moore–Penrose principle. If *N* > *L*, the optimal solution of equation (3) is:

(5) $$\begin{array}{c} \beta^{*}=\left(H^{T}H+\frac{I_{L}}{\theta }\right)H^{T}\mathrm{Y,} \end{array}$$

where **I**_*L*_ is a *L*-dimensional unit matrix.

If *N* ≤ *L*, the optimal solution of equation (3) is:

(6) $$\begin{array}{c} \beta^{*}=H^{T}\left(H^{T}H+\frac{I_{N}}{\theta }\right)Y, \end{array}$$

where **I**_*N*_ is an *N*-dimensional unit matrix.

## 3. Proposed Methods

In this section, the overall architecture of the proposed TSTELM is introduced in detail. As shown in Figure 1, TSTELM consists of three parts: statistical matching stage, subspace alignment stage, and prediction based on weight fusion.

### 3.1. Statistical Matching Stage

In statistical matching stage, we hope to obtain an ELM for domain adaptation using labeled samples of the source domain and unlabeled samples of the target domain. First, the source data and target data are mapped into the hidden layer space of ELM, and then we could obtain **H**_*S*_={(**h**_*Si*_, **y**_*i*_)}_*i*=1_^*n*_*S*_^ and **H**_*T*_={(**h**_*Tj*_)}_*j*=1_^*n*_*T*_^, respectively, where *h*_*S*_(*x*_*i*_)=*g*(**w***x*_*Si*_+**b**) and *h*_*T*_(*x*_*j*_)=*g*(**w***x*_*Tj*_+**b**), *n*=*n*_*S*_+*n*_*T*_, **w** ∈ *R*^*d*×*L*^ and **b** ∈ *R*^1×*L*^ are randomly generated weights and bias, *d* is the original spatial dimension of the data.

For labeled source data, we can learn an ELM, that is

(7) $$\begin{array}{c} \underset{\beta_{S}}{\text{min}}:\frac{1}{2}{\left\|\beta_{S}\right\|}^{2}+\frac{1}{2}{\left\|H_{S}\beta_{S}-Y_{S}\right\|}^{2}, \end{array}$$

where *β*_*S*_ is the output weight of the ELM learned on {**H**_*S*_, **Y**_*S*_}. Since equation (7) just obtain an ELM classifier using the labeled source samples, it cannot perform well for the target domains due to distribution difference between the source and target domains. Therefore, we adopt MMD between **H**_*S*_ and **H**_*T*_ to reduce marginal and conditional distribution difference between domains [42]. MMD minimization is formulated as:

(8) $$\begin{array}{c} \text{MMD}\left(\beta \right)=\underset{\beta }{\min}{\left\|\frac{1}{n_{S}}\sum_{i=1}^{n_{S}}h\left(x_{i}\right)\beta -\frac{1}{n_{T}}\sum_{j=1}^{n_{T}}h\left(x_{j}\right)\beta \right\|}_{ℋ}^{2}+\sum_{c=1}^{C}{\left\|\frac{1}{n_{S}^{\left(c\right)}}\sum_{x_{i}\in D_{S}^{\left(c\right)}}h\left(x_{i}^{\left(c\right)}\right)\beta -\frac{1}{n_{T}^{\left(c\right)}}\sum_{x_{j}\in D_{T}^{\left(c\right)}}h\left(x_{j}^{\left(c\right)}\right)\beta \right\|}_{ℋ}^{2}\\ =\underset{\beta }{\text{min}}\text{tr}\left(\beta^{T}H^{T}\left(M_{0}+\sum_{c=1}^{C}M_{c}\right)\mathrm{H\beta}\right), \end{array}$$

where **H**=**H**_*S*_^T^ ∪ **H**_*T*_^T^; **M**_0_ and **M**_*c*_ are the MMD matrixes which are as follows:

(9) $$\begin{array}{c} {\left(M_{0}\right)}_{ij}=\left\{\begin{array}{cc} \frac{1}{n_{S}n_{S}}, & x_{i},x_{j}\in D_{S},\\ \frac{1}{n_{T}n_{T}}, & x_{i},x_{j}\in D_{T},\\ \frac{-1}{n_{S}n_{T}}, & \text{otherwise,} \end{array}\right. \end{array}$$

(10) $$\begin{array}{c} {\left(M_{c}\right)}_{ij}=\left\{\begin{array}{cc} \frac{1}{n_{S}^{\left(c\right)}n_{S}^{\left(c\right)}}, & x_{i}^{\left(c\right)},x_{j}^{\left(c\right)}\in D_{S}^{\left(c\right)},\\ \frac{1}{n_{T}^{\left(c\right)}n_{T}^{\left(c\right)}}, & x_{i}^{\left(c\right)},x_{j}^{\left(c\right)}\in D_{T}^{\left(c\right)},\\ \frac{-1}{n_{S}^{\left(c\right)}n_{T}^{\left(c\right)}}, & \left\{\begin{array}{c} x_{i}^{\left(c\right)}\in D_{S}^{\left(c\right)}\text{and}x_{j}^{\left(c\right)}\in D_{T}^{\left(c\right)},\\ x_{j}^{\left(c\right)}\in D_{S}^{\left(c\right)}\text{and}x_{i}^{\left(c\right)}\in D_{T}^{\left(c\right)}, \end{array}\right.\\ 0, & \text{otherwise,} \end{array}\right. \end{array}$$

where **D**_*S*_^(*c*)^ and **D**_*T*_^(*c*)^ are the sample subsets with label category *c* in the source and target domains; **x**_*i*_^(*c*)^ and **x**_*j*_^(*c*)^ are the samples in **D**_*S*_^(*c*)^ and **D**_*T*_^(*c*)^, respectively; *n*_*S*_^(*c*)^ and *n*_*T*_^(*c*)^ are the number of samples in **D**_*S*_^(*c*)^ and **D**_*T*_^(*c*)^, respectively.

Here, replacing *β*_*S*_ and *β* with *β*_1_ and incorporating equations (7) and (8), we can obtain the DAELM at statistical matching stage, and its objective function is

(11) $$\begin{array}{c} \underset{\beta }{\min}\frac{1}{2}{\left\|\beta_{1}\right\|}^{2}+\frac{\theta }{2}{\left\|H_{S}\beta_{1}-Y_{S}\right\|}^{2}+\frac{\lambda }{2}\mathrm{Tr}\left(\beta_{1}^{T}H^{T}\left(M_{0}+\sum_{c=1}^{C}M_{c}\right)H\beta_{1}\right). \end{array}$$

By setting the gradient of equation (11) with respect to *β*_1_ as zero, we have

(12) $$\begin{array}{c} \beta_{1}=\left\{\begin{array}{cc} H^{T}{\left(\mathrm{HE}H^{T}+\lambda \left(M_{0}+\sum_{c=1}^{C}M_{c}\right)HH^{T}+\frac{I_{L}}{\theta }\right)}^{-1}EY_{S}^{T}, & n>L,\\ {\left(H^{T}\mathrm{EH}+\lambda H^{T}\left(M_{0}+\sum_{c=1}^{C}M_{c}\right)H+\frac{I_{n}}{\theta }\right)}^{-1}H^{T}EY_{S}^{T}, & n\leq L, \end{array}\right. \end{array}$$

where **E** is a diagonal label indicator matrix with each element *E*_*ii*_=1 if **x**_*i*_ ∈ **D**_*S*_, and *E*_*ii*_=0 otherwise.

### 3.2. Subspace Alignment Stage

At subspace alignment stage, we train a DAELM on labeled samples of the source domains and unlabeled samples of the target domains.

For the target sample, we can learn an ELM from the following formula:

(13) $$\begin{array}{c} \underset{\beta_{T}}{\text{min}}:\frac{1}{2}{\left\|\beta_{T}\right\|}^{2}+\frac{\alpha }{2}{\left\|H_{T}\beta_{T}-H_{S\_av}\beta_{1}\right\|}^{2}+\frac{\alpha }{2}\sum_{c=1}^{C}{\left\|H_{T}^{\left(c\right)}\beta_{T}-H_{S\_av}^{\left(c\right)}\beta_{1}\right\|}^{2},\\ \Leftrightarrow \underset{\beta_{T}}{\min}:\frac{1}{2}{\left\|\beta_{T}\right\|}^{2}+\frac{\alpha }{2}\sum_{c=0}^{C}{\left\|H_{T}^{\left(c\right)}\beta_{T}-H_{S\_av}^{\left(c\right)}\beta_{1}\right\|}^{2}. \end{array}$$

Here, inspired by [35], we introduce cross-domain mean approximation to replace the prediction loss. When there are no labeled samples in the target domains (when *c*=0), we force target data **H**_*T*_ close to source data mean point **H**_*S*_*av*_, which promotes domain adaptation seen from [35]. If the target sample obtains pseudo labels, it is drawn to source data mean point with the same category **H**_*S*_*av*_^(*c*)^.

In order to further improve cross-domain knowledge transferring, similar to [38], we introduce a transformation matrix **M** to align the output weights of ELM between the source domain and the target domain. The function is established as follows:

(14) $$\begin{array}{c} f\left(M\right)=\min{\left\|\beta_{1}M-\beta_{T}\right\|}_{F}^{2}, \end{array}$$

where ‖•‖_*F*_^2^ is Frobenius norm. It is invariant to the orthogonalization operation, so equation (14) can be rewritten as:

(15) $$\begin{array}{c} f\left(M\right)=\min{\left\|\beta_{1}^{T}\beta_{1}M-\beta_{1}^{T}\beta_{T}\right\|}_{F}^{2}\\ =\min{\left\|M-\beta_{1}^{T}\beta_{T}\right\|}_{F}^{2}. \end{array}$$

Then, we can get the optimal **M***∗*=*β*_1_^*T*^*β*_*T*_. Let *β*_*a*_=*β*_1_**M**=*β*_1_*β*_1_^*T*^*β*_*T*_, we can know that *β*_*a*_ is closer to *β*_*T*_ than *β*_1_ and facilitates cross-domain knowledge transfer.

To align output layer of source ELM to target one, we combine the training error ‖**H**_*S*_*β*_*a*_ − **Y**_*S*_‖^2^, equation (13), and a regular term and replace *β*_1_ with *β*_*a*_ to get:

(16) $$\begin{array}{c} J\left(\beta_{a},\beta_{T}\right)=\underset{\beta_{a},\beta_{T}}{\min}\frac{1}{2}{\left\|\beta_{T}\right\|}^{2}+\frac{\theta }{2}{\left\|H_{S}\beta_{a}-Y_{S}\right\|}^{2}+\frac{\alpha }{2}\sum_{c=0}^{C}{\left\|H_{T}^{\left(c\right)}\beta_{T}-H_{S\_av}^{\left(c\right)}\beta_{1}\right\|}^{2}+\frac{1}{2}{\left\|\beta_{T}-\beta_{a}\right\|}^{2}, \end{array}$$

where ‖*β*_*T*_ − *β*_*a*_‖^2^ is a parameter approximation term for facilitating knowledge transfer and preventing negative transfer, and *λ* and *γ* are the balance parametesr. We substitute *β*_*a*_=*β*_1_*β*_1_^T^*β*_*T*_ to equation (16) and get:

(17) $$\begin{array}{c} J\left(\beta_{T}\right)=\underset{\beta_{T}}{\min}\frac{1}{2}{\left\|\beta_{T}\right\|}^{2}+\frac{\theta }{2}{\left\|H_{S}\beta_{1}\beta_{1}^{T}\beta_{T}-Y_{S}\right\|}^{2}+\frac{\alpha }{2}\sum_{c=0}^{C}{\left\|H_{T}^{\left(c\right)}\beta_{T}-H_{S\_av}^{\left(c\right)}\beta_{1}\right\|}^{2}+\frac{1}{2}{\left\|\beta_{T}-\beta_{1}\beta_{1}^{T}\beta_{T}\right\|}^{2}\\ =\underset{\beta_{T}}{\min}\frac{1}{2}{\left\|\beta_{T}\right\|}^{2}+\frac{\theta }{2}{\left\|H_{S}\beta_{1}\beta_{1}^{T}\beta_{T}-Y_{S}\right\|}^{2}+\frac{\alpha }{2}\sum_{c=0}^{C}{\left\|H_{T}^{\left(c\right)}\beta_{T}-H_{S\_av}^{\left(c\right)}\beta_{1}\right\|}^{2}+\frac{1}{2}{\left\|\left(I-\beta_{1}\beta_{1}^{T}\right)\beta_{T}\right\|}^{2}. \end{array}$$

Because ‖(**I** − *β*_1_*β*_1_^T^)*β*_*T*_‖^2^ ≤ ‖(**I** − *β*_1_*β*_1_^T^)‖^2^‖*β*_*T*_‖^2^, we change equation (17) into:

(18) $$\begin{array}{c} J\left(\beta_{T}\right)\\ =\underset{\beta_{T}}{\min}\frac{1}{2}{\left\|\beta_{T}\right\|}^{2}+\frac{\theta }{2}{\left\|H_{S}\beta_{1}\beta_{1}^{T}\beta_{T}-Y_{S}\right\|}^{2}+\frac{\alpha }{2}\sum_{c=0}^{C}{\left\|H_{T}^{\left(c\right)}\beta_{T}-H_{S\_av}^{\left(c\right)}\beta_{1}\right\|}^{2}+\frac{1}{2}{\left\|\left(I-\beta_{1}\beta_{1}^{T}\right)\right\|}^{2}{\left\|\beta_{T}\right\|}^{2}\\ =\underset{\beta_{T}}{\min}\frac{1}{2}{\left\|\left(\begin{array}{c} \theta H_{S}\beta_{1}\beta_{1}^{T}\\ \alpha H_{T} \end{array}\right)\beta_{T}-\left(\begin{array}{c} Y_{S}\\ \alpha \sum_{c=0}^{C}H_{S\_av}^{\left(c\right)}\beta_{1} \end{array}\right)\right\|}^{2}+\frac{\left(I+{\left(I-\beta_{1}\beta_{1}^{T}\right)}^{T}\left(I-\beta_{1}\beta_{1}^{T}\right)\right)}{2}{\left\|\beta_{T}\right\|}^{2}. \end{array}$$

Let $Q=\left(\begin{array}{c} \theta H_{S}\beta_{1}\beta_{1}^{T}\\ \alpha H_{T} \end{array}\right),T=\left(\begin{array}{c} Y_{S}\\ \alpha \sum_{c=0}^{C}H_{S\_av}^{\left(c\right)}\beta_{1} \end{array}\right),\text{ and }A=I+{\left(I-\beta_{1}\beta_{1}^{T}\right)}^{T}\left(I-\beta_{1}\beta_{1}^{T}\right),$ and equation (18) can be simplified as

(19) $$\begin{array}{c} J\left(\beta_{T}\right)=\underset{\beta_{T}}{\min}:\frac{1}{2}{\left\|Q\beta_{T}-T\right\|}^{2}+\frac{A}{2}{\left\|\beta_{T}\right\|}^{2}. \end{array}$$

Then:

(20) $$\begin{array}{c} \beta_{2}=\beta_{T}^{*}=\left\{\begin{array}{cc} {\left(Q^{T}Q+A\right)}^{-1}Q^{T}T, & n>L,I\text{ in}A\text{ is an }L-\text{dimensional unit matrix,}\\ Q^{T}{\left(QQ^{T}+A\right)}^{-1}T, & n\leq L,I\text{ in}A\text{ is an }n-\text{dimensional unit matrix}. \end{array}\right. \end{array}$$

### 3.3. Prediction Based on Output Weight Fusion

In the classification task, a sample **x**_*Te*_ is tested. After *β*_1_ and *β*_2_ are obtained, the output weight of final ELM model is dominated by *β*^*∗*^=*β*_2_+*pβ*_1_, and the classification result of **x**_*Te*_ can be obtained:

(21) $$\begin{array}{c} y_{Te}=\left\{\begin{array}{cc} \text{sign}\left(h_{Te}^{T}\beta^{*}\right), & \text{for binary classification},\\ \text{argmax}\left(h_{Te}^{T}\beta^{*}\right), & \text{for multi}-\text{class classification,} \end{array}\right. \end{array}$$

where **h**_*Te*_=*g*(**x**_*Te*_) and *p* is the scale factor to balance *β*_1_ and *β*_2_.

TSTELM can be summarized in Algorithm 1.

### 3.4. Discussion

In order to solve the problem that the traditional ELM does not perform well in cross-domain tasks, we propose TSTELM and its objective function is equations (8) and (17). It can be seen:

1. Compared with the classical ELM, TSTELM reduces the distribution difference between domains and transfers knowledge across domains via adopting MMD, output weight alignment, parameter approximation, and ∑_*c*=0_^*C*^‖**H**_*T*_^(*c*)^*β*_*T*_ − **H**_*S*_*av*_^(*c*)^*β*_1_‖^2^.
2. Though TELM-OWA proposed by Zang et al. [38] also applies output weight alignment and parameter approximation for domain adaptation, it is a supervised domain adaptation algorithm requiring few target labeled samples unlike TSTELM. In addition, TSTELM replaces ‖**H**_*T*_*β*_*T*_ − **Y**_*T*_‖^2^ with ∑_*c*=0_^*C*^‖**H**_*T*_^(*c*)^*β*_*T*_ − **H**_*S*_*av*_^(*c*)^*β*_1_‖^2^, which is different from TELM-OWA.
3. Different from DAELM-S, DAELM-T, TELM-OWA, and CDELM, in which only one output weight *β*^*∗*^ is solved, our method needs the learned weights of two stages to fuse and then make decisions, which shows that TSTELM has strong robustness similar to ensemble learning.
4. In domain adaptation, we consider samples from the source domains as training datasets and samples from the target domains as testing datasets, so the output matrixes **H**_*S*_ and **H**_*T*_ are computed which have time complexity of *O*(*Ln*_*S*_*d*) and *O*(*Ln*_*T*_*d*). The main time cost of ELM is equation (5) or (6), and the time complexity is:

(22) $$\begin{array}{c} \text{O}\left(n_{S}^{3}+2Ln_{S}^{2}+mLn_{S}\right)\text{when,}n_{S}<\mathrm{L,}\\ \text{O}\left(L^{3}+L^{2}n_{S}+m{\text{Ln}}_{S}\right)\text{when,}n_{S}>L. \end{array}$$

According to Algorithm 1, the main computation cost of our method is in steps 3 and 4.

In step 3, we need to compute **M**_0_, ∑_*c*=1_^*C*^**M**_*c*_, (**E**+**M**_0_+∑_*c*=1_^*C*^**M**_*c*_)**HH**^T^, **H**^T^(**E**+**M**_0_+∑_*c*=1_^*C*^**M**_*c*_)**H**, the inverse of matrix with *N* × *N* or *L* × *L* size and **H**^T^**EY**_*S*_ which has time complexity *O*(*N*^2^), *O*(*CN*^2^), *O*(*N*^3^*+LN*^*2*^), *O*(*LN*^*2*^+*L*^*2*^*N*), *O*(*N*^3^) or *O*(*L*^3^), and *O*(CLN*+LN*^*2*^). Therefore, the time complexity of step 2 is

(23) $$\begin{array}{c} O\left(2{\text{TN}}^{3}+2{\text{TLN}}^{2}+T\left(C+1\right)N^{2}+\text{TCLN}\right)\text{when,}N<\mathrm{L,}\\ O\left({\text{TL}}^{3}+2{\text{TLN}}^{2}+{\text{TL}}^{2}N+T\left(C+1\right)N^{2}+\text{TCLN}\right)\text{when,}N>\mathrm{L,} \end{array}$$

where *T* is the number of iterations.

In step 4, the output weight is determined according to equation (20) and **Q** has the same size of **H**. Therefore, the time complexity of step 4 is:

(24) $$\begin{array}{c} \text{O}\left(TN^{3}{+2\text{TLN}}^{2}+\text{TCLN}\right)\text{when,}N<\mathrm{L,}\\ \text{O}\left(TL^{3}+TL^{2}N+\text{TCLN}\right)\text{when,}N>L. \end{array}$$

Given that TELM-OWA also has two stages to compute the output weight, it has time complexity in the first stage as follows:

(25) $$\begin{array}{c} \text{O}\left(n_{S}^{3}+2Ln_{S}^{2}{+\text{mLn}}_{S}\right)\text{when,}n_{S}<\mathrm{L,}\\ \text{O}\left(L^{3}+L^{2}n_{S}{+\text{mLn}}_{S}\right)\text{when,}n_{S}>L. \end{array}$$

The time complexity of TELM-OWA in the second stage is

(26) $$\begin{array}{c} \text{O}\left(N^{3}+2LN^{2}+\text{CLN}\right)\text{when,}N<\mathrm{L,}\\ \text{O}\left(L^{3}+L^{2}N+\text{CLN}\right)\text{when,}N>L. \end{array}$$

The above analysis indicates that the computational complexity of TSTELM is significantly higher than ELM and TELM-OWA.

## 4. Experiment and Analysis

In this section, experiments are conducted on four cross-domain datasets including Office + Caltech object recognition, USPS and MNIST digital handwriting, MSRC and VOC2007 object recognition, and Reuters-21578 text dataset for classification, where image datasets are descripted in Table 2. We compare our approach with several related unsupervised classification methods and semi-supervised and unsupervised domain adaptation methods. To be more objective, experiments are implemented on PC with 8 GB memory and Windows 10 operating system and MATLAB 2017b. Every experiment runs 20 times and the average value is recorded. We adopt the accuracy rate to evaluate the performance of every algorithm, and it is

(27) $$\begin{array}{c} \text{Accuracy}=\frac{\text{correctly\_classified\_samples}}{\text{total\_samples}}\times 100\%. \end{array}$$

### 4.1. Dataset Description

*aOffice* *+* *Caltech256* (shown in Figure 3): Office is widely used dataset for visual cross-domain learning, which contains 4,652 images in 31 categories. These images come from 3 realistic aggregated item datasets: Amazon (images download from online chants https://www.amazon.com); DSLR (high-resolution images by a digital SLR camera in realistic environments); and Webcam (low-resolutions images by a simple webcam). Caltech256 is also a standard object recognition dataset which contains 30,607 images from 256 categories.

In this article, we employ the Office + Caltech dataset released by Gong et al. [57]. SURF features are extracted and quantized into an 800-bin histogram with codebooks computed with K-means on a subset of images from Amazon. Then, the histograms are standardized by z-score. We select four domains C (Caltech256), A (Amazon), W (Webcam), and D (DSLR) for experiment, and two different domains are randomly selected as the source and the target domain datasets, and 12 cross-domain tasks for evaluation are constructed, namely C ⟶ A, C ⟶ W, C ⟶ D,…, and D ⟶ W.

*USPS* *+* *MNIST* (as shown in Figure 4): USPS and MNIST are the two different but related handwritten datasets with 10 categories of 0–9. The USPS dataset contains 7,291 training samples and 2,007 test samples with 16 × 16 pixels. There are 60,000 training images and 10,000 test images with 28 × 28 pixels in the MNIST database.

During this experiment, we randomly select 1,800 pictures from USPS and 2,000 pictures from MNIST and convert them into 16 × 16 pixels. We construct two cross-domain tasks, that is USPS as the source domain and MNIST as the target domain (USPS vs MNIST) and vice versa (MNIST vs USPS).

*MSRC* *+* *VOC2007* (shown in Figure 5): MSRC dataset is provided by Microsoft Cambridge, which consists of 4323 images of 18 object classes. VOC2007 dataset contains 5,011 images annotated with 20 concepts. We can see from Figure 5 that MSRC and VOC2007 have distinct but different distributions. MSRC are standard images as benchmark data for evaluation. VOC2007 is randomly constructed by using the images in the network album.

In our experiments, we construct the domain adaptation dataset MSRC vs VOC in which 6 shared categories are selected including aircraft, birds, cows, family cars, sheep and bicycles. Among them, 1269 images are selected from the MSRC dataset as the source domain dataset and 1530 images are selected from the VOC2007 dataset as the target domain dataset. Then, the source domain and the target domain are exchanged to construct a new set of domain adaptation dataset VOC vs MSRC. We convert all images into 256 gray pixels; 240 dimensions are extracted as the spatial dimension of the sample.

*Reuters-21578*: Reuters-21578 text dataset is a common dataset for text classification. It contains 21,577 news documents from Reuters in 1987. These documents have been manually labeled by Reuters as five classes, such as “exchanges,” “orgs,” “people,” “places,” and “topics,” including multiple categories and subclasses. Among them, the largest three categories are “orgs,” “people,” and “place,” which can construct six cross-domain text classification tasks orgs vs people, people vs orgs, orgs vs place, place vs orgs, people vs place, and place vs people. This article makes a more complete evaluation of the algorithm on 6 classification tasks.

### 4.2. Experimental Settings

To validate the efficiency of TSTELM, we compare it with some other classifiers.

*Classifiers for non-domain adaptation*: 1NN, SVM, ELM, and SSELM [58] (ELM with graph regularization term for semi-supervised learning).

*Classifiers for domain adaptation*: TCA1 [47](TCA with 1NN for classification), TCA2 [47] (TCA with SVM for classification), JDA1 [48] (JDA with 1NN for classification), JDA2 [48](JDA with SVM for classification), DAELM-S [36], DAELM-T [36], ARRLS [59], TELM-OWA [38], JPDA [60], AELM [61], DST-ELM [40], CDELM [39], and TSTELM.

In order to achieve the optimal performance of each algorithm in the experiment, we set SVM penalty parameter belonging to {0.1, 0.5, 1,5,10,50,100}, and the penalty parameter *θ* ∈ [0.001, 0.1] in ELM, SSELM, DAELM_S, DAELM_T, TELM-OWA, and TSTELM. TCA(1,2) and JDA(1,2) are combined feature extraction with standard classifier for domain adaptation, in which the dimension of the feature subspace is 100 and the value range of the balanced-constraint parameter of the projection matrix in TCA and JDA is [0.1, 1]. The parameters of ARRLS, DAELM_S, DAELM_T, and TELM-OWA are set according to the corresponding literature. In TSTELM, we set *α* ∈ [10^3^, 10^4^], *λ* ∈ [10^−3^, 10^−4^],and *L*=1500 on Office + Caltech dataset, *L*=3000 on USPS + MNIST and MSRC + VOC2007 datasets, *L*=5000 on Reuters-21578 dataset. We cite results of JPDA, AELM, DST-ELM, and CDELM from those corresponding literature.

In fact, DAELM_S, DAELM_T, and TELM-OWA, as supervised models, need a few labeled target samples to induce the target classifier. We test them with 0.5% labeled target samples on USPS + MNIST, MSRC + VOC2007, and Reuters-21578 datasets and 1% labeled target samples on Office + Caltech dataset, to approximate the performance of these methods in unsupervised domain adaptation.

### 4.3. Experimental Results and Analysis

We test TSTELM on Office + Caltech256, USPS + MNIST, MSRC + VOC2007, and Reuters-21578 datasets, and the comparison results are displayed in Tables 3 and 4 and Figures 4–8, in which the best results of each task are bold. From the comparison of results, we have the following observations.

1. The total average accuracy of TSTELM across 22 tasks is the highest among all methods, indicating that our approach can effectively deal with domain adaptation problem.
2. In unsupervised domain adaptation, the proposed method outperforms AELM, DST-ELM, CDELM, TELM-OWA, DAELM_S, and DAELM_T, indicating the superiority of TSTELM in which MMD and output weight alignment are unified into the ELM learning framework to minimize distribution discrepancy between domains. AELM, DAELM_S, and DAELM_T obtain poor results, showing that they are highly dependent on labeled target samples. 1NN, SVM, and ELM perform unsuccessfully because of the problem of domain shift. SSELM performs better than ELM due to that the original geometry information of data is mined.
3. TCA(1,2), JDA(1,2), and JPDA are better than 1NN and SVM, showing the importance of shared feature extraction across domains. JPDA and JDA(1,2) are generally higher than TCA(1,2), which indicates the superiority of simultaneously reducing the marginal and conditional distribution discrepancy. ARRLS performs well because of MMD and preserves the manifold consistency at the same time.

We check the execution times of some methods on MNIST vs USPS, and the results are reported in Table 5. It can be seen: (1) The speed of the methods based on ELM are significantly faster than other methods, and ELM is the fastest. (2) TSTELM consumes more time than TELM-OWA, ELM, SSELM, DAELM_S, and DAELM_T, because of label refinement iterative process. TELM-OWA is more time-consuming than ELM, SSELM, DAELM_S, and DAELM_T as a result of solving *β*_*S*_^*∗*^ and *β*_*T*_^*∗*^. (3) Since constructing the Laplacian matrix is the most time-consuming, SSELM is relatively inefficient. (4) TCA(1,2) and JDA(1,2) cost more time than 1NN and SVM because of additional feature extraction process. (5) JDA(1,2) has the highest time cost because it applies an iterative manner to refine the target pseudo label and extract cross-domain shared feature.

### 4.4. Parameter Analysis

To evaluate the effects of scale factor (*p*); number of hidden layer nodes(*L*); parameter *α*, *λ*, and *θ* on TSTELM, we conduct some experiments on org vs people, MSRC vs VOC, MNIST vs USPS, and A vs D. The results are shown in Figures 9(a)–9(f). It can be seen that: (1) With the increase of *p*, the trend in TSTELM accuracy goes up first and then goes down on all test datasets and achieves optimal results when *p* ∈ [0.1, 1], as shown in Figure 9(a). It can be known that the results of joint decision of *β*_1_ and *β*_2_ are better than their separate decisions. (2) As shown in Figure 9(b), TSTELM accuracy increases first and then decreases with the number of *L* on all test datasets. Although a large network forces the ELM network to behave better on output function approximation, time cost of the algorithm and required memory become large, and too many hidden nodes will hurt the ELM performance of domain adaptation because of better output function approximation. (3) In Figures 9(c)–9(e), with the gradual increase of parameter *α*, *λ*, and *θ*, the accuracy increases first and then decreases and takes different optimal values on different test datasets to achieve the optimal accuracy, which indicates that the control term of these parameters are beneficial to TSTELM when the parameter values are reasonable. (4) We also provide the classification accuracy varying with the iteration number, and result is shown in Figure 9(f). It shows that the accuracy is increasing iterative with the number of iterations and finally converges after several iterations, which verifies that TSTELM has strong robustness.

## 5. Conclusion

To handle the problem that traditional ELM does not perform well in unsupervised domain adaptation, we in this article propose TSTELM including two domain adaptation stages. At the statistical matching stage, MMD is introduced into ELM learning frame to simultaneously minimize the marginal and conditional distribution between domains. At the subspace alignment stage, subspace alignment strategy, cross-domain mean approximation, and output weight approximation are adopted to further adjust the distribution consistency between domains. Finally, parameters of learned ELM models at two stages are fused and used to predict test samples. Extensive experiments have been conducted on real-world image and text datasets, and the results show that TSTELM has higher accuracy and better generalization performance. In the future, we will make further research that TSTELM is improved by stacking it into deep structure model for extracting deep feature.

## Figures and Tables

**Figure 1:** An illustration of TSTELM. (1) At the statistical matching domain adaptation stage, we use the MMD to simultaneously minimize the marginal and conditional distribution between domains in output layers and get a DAELM. (2) At the subspace alignment domain adaptation stage, we align the output weights of source and target ELM model, simultaneously design target cross-domain mean approximation term, and add the output weight approximation term into the objective function. We can obtain the other DAELM. (3) In fusion decision, we fuse the DAELM parameters from two stages to realize the label prediction of test samples.

**Figure 2:** The structure of ELM.

**Figure 3:** Image samples from (b) Amazon, (d) Caltech256, (a) DSLR, and (c) Webcam.

**Figure 4:** Image samples from (a) MNIST and (b) USPS.

**Figure 5:** Image samples from (a) MSRC and (b) VOC2007.

**Figure 6:** Classification accuracy of different algorithms on (a) USPS + MNIST and (b) MSRC + VOC2007 dataset.

**Figure 7:** Classification accuracy of different algorithms on Office + Caltech256 dataset.

**Figure 8:** Classification accuracy of different algorithms on Reuters-21578 dataset.

**Figure 9:** Classification accuracy of TSTELM with respect to scale factor (*p*); number of hidden layer nodes (*L*); parameter *α*, *λ*, and *θ*; and iteration.

**Algorithm 1:** TSTELM.

**Table 1:** Notations.

Terminology	Source	Target
Domain	**D**_*S*_={*𝒳*_*S*_, *P*(**X**_*S*_)}	**D**_*T*_={*𝒳*_*T*_, *P*(**X**_*T*_)}
Data	**X**_*S*_={(**x**_*Si*_, **y**_*i*_)}_*i*=1_^*n*_*S*_^	**X**_*T*_={(**x**_*Tj*_)}_*j*=1_^*n*_*T*_^
Feature space	*𝒳*_*S*_	*𝒳*_*T*_
Label space	*𝒴*_*S*_	*𝒴*_*T*_
Marginal distribution	*P*_*S*_(**X**_*S*_)	*P*_*T*_(**X**_*T*_)
Conditional distribution	*P*(**Y**_*S*_*| ***X**_*S*_)	*P*(**Y**_*T*_*| ***X**_*T*_)
Task	**T**_*S*_={*𝒴*_*S*_, *P*(**Y**_*S*_*| ***X**_*S*_)}	**T**_*T*_={*𝒴*_*T*_, *P*(**Y**_*T*_*| ***X**_*T*_)}

**Table 2:** Description of image dataset.

Dataset	Type	Samples	Dimension	Class	Contains subsets
USPS	Digit	1800	256	10	USPS
MNIST	Digit	2000	256	10	MNIST
MSRC	Object	1269	240	18	MSRC
VOC2007	Object	1530	240	20	VOC
Office	Object	1410	800	10	A, W, D
Caltech	Object	1123	800	10	C

**Table 3:** Accuracy of different algorithms on Office + Caltech256 and USPS + MNIST datasets.

Methods	Dataset																
	C ⟶ A(1)	C ⟶ W(2)	C ⟶ D(3)	A ⟶ C(4)	A ⟶ W(5)	A ⟶ D (6)	W ⟶ C (7)	W ⟶ A (8)	W ⟶ D(9)	D ⟶ C(10)	D ⟶ A(11)	D ⟶ W(12)	Average	USPS vs MNIST	MNIST vs USPS	Average	Total average
1NN	23.70	25.76	25.48	26.00	29.83	25.48	19.86	22.96	59.24	26.27	28.50	63.39	31.37	44.70	65.94	55.32	34.79
SVM	52.40	40.68	42.04	44.08	41.69	40.76	29.92	34.13	**87.90**	31.43	32.36	73.56	45.91	35.10	54.69	44.9	45.77
ELM	50.63	42.71	42.04	43.01	37.63	42.68	32.24	36.85	80.25	30.10	31.52	71.86	45.13	30.70	51.39	41.05	44.54
SSELM	52.92	45.42	38.85	41.76	35.93	38.85	34.28	37.06	78.98	30.37	32.05	80.00	45.54	29.05	43.28	36.16	44.2
TCA1	55.85	48.81	**51.59**	44.17	40.34	36.94	32.32	38.41	81.53	36.24	39.35	82.37	48.99	35.55	53.34	44.45	48.34
TCA2	55.01	48.48	49.68	**44.35**	41.02	43.31	32.59	38.94	79.62	34.64	38.31	**83.89**	49.15	34.70	52.78	43.74	48.38
JDA1	53.34	46.78	52.87	42.65	36.27	40.76	33.66	47.60	86.89	36.51	43.31	82.73	47.33	34.77	54.92	44.85	49.5
JDA2	54.80	51.86	51.22	41.23	39.66	44.59	35.09	45.51	80.26	33.39	40.92	83.05	50.13	33.86	53.11	43.49	49.18
DAELM_S	50.26	45.42	37.58	42.88	38.31	36.94	34.20	36.44	80.89	32.32	34.35	72.88	45.21	44.36	47.11	45.73	45.28
DAELM_T	27.85	31.86	22.93	25.25	19.32	36.31	**41.90**	**46.49**	53.50	**48.08**	**51.20**	54.24	38.24	31.08	60.32	45.7	39.31
ARRLS	54.91	50.51	44.59	42.48	38.98	38.85	34.73	39.87	78.34	32.24	37.16	82.71	47.95	34.64	52.48	43.56	47.32
JPDA	47.60	45.76	46.5	40.78	40.68	36.94	34.55	33.82	88.54	34.73	34.66	91.19	47.98	59.2	68.94	**64.07**	50.28
AELM	52.40	43.73	47.77	40.16	34.92	35.67	30.54	37.16	86.62	28.67	29.54	83.73	45.91	41.65	62.83	52.24	46.81
DST-ELM (mar)	51.88	46.1	44.59	43.72	44.41	40.13	33.93	36.22	74.52	32.06	34.45	77.97	46.67	43.9	59.83	51.87	47.41
DST-ELM (con)	53.65	**51.53**	49.04	37.49	39.66	**50.96**	35.98	42.07	82.17	29.47	44.05	84.07	50.01	50.85	**73.39**	62.12	51.74
CDELM-M	52.07	51.05	45.86	42.33	42.85	45.86	30.31	39.83	81.15	30.31	35.72	81.76	48.26	46.53	62.47	54.5	49.15
CDELM-C	**56.28**	50.98	43.82	43.17	40.75	41.78	34.44	39.58	83.06	34.44	39.54	84.34	49.35	45.89	42.57	44.23	48.62
TELM-OWA	31.73	32.20	33.12	38.85	38.64	43.31	33.48	38.01	77.07	32.50	36.23	78.64	42.82	**59.55**	59.37	59.46	45.19
TSTELM	56.26	50.47	49.1	42.27	**44.75**	47.22	35.26	39.24	78.34	35.44	40.29	83.38	**50.17**	58.55	69.44	62.96	**52.86**

The bold values in Table 3 is best result in its column.

**Table 4:** Accuracy of different algorithms on MSRC + VOC2007 and Reuters-21578 datasets.

Methods\dataset	Non-transfer learning algorithm				Transfer learning algorithm								
	1NN	SVM	ELM	SSELM	TCA1	TCA2	JDA1	JDA2	DAELM_S	DAELM_T	ARRLS	TELM-OWA	TSTELM
MSRC vs VOC	35.95	35.10	38.56	37.52	27.91	34.90	27.12	34.77	38.34	33.60	34.64	**41.37**	36.47
VOC vs MSRC	45.23	54.69	58.00	63.20	47.91	54.22	48.31	54.61	58.37	30.61	50.35	66.22	**75.23**
*Average*	40.59	44.90	48.28	50.36	37.91	44.56	37.71	44.69	48.35	32.10	42.50	53.79	**55.85**
Orgs vs people (1)	72.85	75.25	77.24	80.30	76.49	77.51	80.13	81.79	76.64	48.71	80.55	63.74	**83.27**
People vs orgs (2)	72.03	77.12	79.30	84.72	77.28	79.39	85.13	85.29	78.41	47.72	84.56	64.27	**85.69**
Orgs vs place (3)	67.50	70.18	63.57	69.61	72.39	71.81	75.74	**76.22**	68.53	43.81	72.20	68.09	73.92
Place vs orgs (4)	61.12	63.77	64.57	71.16	68.21	65.75	**76.38**	76.08	68.77	42.50	74.11	74.68	73.52
People vs place (5)	52.65	60.63	57.01	66.02	61.19	60.63	**66.85**	65.83	59.14	42.46	65.18	59.04	61.74
Place vs people (6)	53.39	57.94	58.68	61.65	56.08	51.07	58.12	51.16	58.77	39.93	58.56	60.45	**60.81**
*Average*	63.26	67.48	66.73	72.24	68.61	67.69	73.73	72.73	68.38	44.19	72.53	65.05	**73.16**
*Total average*	57.59	61.84	62.12	66.77	60.93	61.91	64.72	65.72	63.37	41.17	65.02	62.23	**68.83**

The bold values in Table 3 is best result in its row.

**Table 5:** Average runtime of all the methods on MNIST vs USPS.

Algorithm	1NN	SVM	ELM	SSELM	TCA1	TCA2	JDA1	JDA2	DAELM_S	DAELM_T	ARRLS	TELM-OWA	TSTELM
Time (s)	0.55	8.79	0.37	3.49	4.72	5.47	48.32	53.6	0.81	0.64	2.08	3.7	36.5

## Data Availability

The data used to support the findings of this study can be found at https://github.com/jindongwang/transferlearning/blob/master/data/dataset.md.
